# A Preliminary Molecular Phylogeny of Planthoppers (Hemiptera: Fulgoroidea) Based on Nuclear and Mitochondrial DNA Sequences

**DOI:** 10.1371/journal.pone.0058400

**Published:** 2013-03-14

**Authors:** Nan Song, Ai-Ping Liang

**Affiliations:** 1 Key Laboratory of Zoological Systematics and Evolution, Institute of Zoology, Chinese Academy of Sciences, Beijing, China; 2 Henan Entry-Exit Inspection and Quarantine Bureau, Zhengzhou, China; University of Sydney, Australia

## Abstract

The planthopper superfamily Fulgoroidea (Insecta: Hemiptera) is one of the most dominant groups of phytophagous insects. It comprises about 20 families, containing a total of 9000 species worldwide. Despite several recent studies, the phylogeny of Fulgoroidea is not yet satisfactorily resolved and the phylogenetic positions of several key families, especially Cixiidae, Delphacidae, Tettigometridae, Nogodinidae, Acanaloniidae and Issidae, are contentious. Here, we expand upon recent phylogenetic work using additional nuclear (*18S* and *28S*) and novel mitochondrial (*16S* and *cytb*) markers. Maximum likelihood and Bayesian analyses yielded robust phylogenetic trees. In these topologies, a group containing Cixiidae and Delphacidae is recovered as the sister group to the remaining taxa. Tettigometridae is placed in a more nested position and is grouped with Caliscelidae. Sister relationships are found between Flatidae and Ricaniidae, and between Dictyopharidae and Fulgoridae. Nogodinidae and Issidae are confirmed to be non-monophyletic families. For major nodes of interest, divergence date estimates are generally older than those from the fossil record.

## Introduction

The planthopper superfamily Fulgoroidea (Insecta: Hemiptera) is among the dominant groups of phytophagous insects, which includes ∼20 families and more than 9000 species worldwide [1]. All species in Fulgoroidea are terraneous and plant-feeding, and many of them are economically significant pests of major agricultural crops such as corn, wheat, rice, and barley. Due to high reproductive potentials and capabilities of transmitting plant pathogens, some delphacid planthoppers have caused substantial damage to grain production and have been identified as the causes for rice famines in several Asian countries for centuries [2]. A number of planthopper species display bizarre morphology (e.g., the elongated head of *Pyrops candelaria*), are brilliantly colored, and some produce cuticular waxes (e.g., the white wax of *Geisha distinctissima*), which make them of considerable interest to biologists. However, the systematic relationships among fulgoroid families remain insufficiently resolved.

Planthoppers are traditionally distinguished from other auchenorrhynchan insects by their antennal sensillae and hind coxae, which are synapomorphies. Muir [3] proposed a grouping for Fulgoroidea by standard morphological characters (e.g., number of tarsal spines) that were considered to be “distinct enough” to warrant familial status, though some of the families as they now stand are also likely to have a polyphyletic origin. The morphological phylogenetic analysis of the Fulgoroidea by Asche [4] led to planthoppers being classified in three major groups, with Tettigometridae as the sister clade to the other fulgoroids, with Cixiidae and Delphacidae grouped together, and with the remaining families in one group. Using 50 adult and nymphal characters, Emeljanov [5] presented a phylogenetic reconstruction of fulgoroids, which was a more fully resolved phylogeny at the family level compared to Asche [4]. Chen and Yang [6] further divided the members of Fulgoroidea into five family-groups on the basis of nymphal traits. The four phylogenetic hypotheses above all supported the sister relationship of Tettigometridae to the other families in Fulgoroidea. In contrast, using morphology of the adult female genitalia, Bourgoin [7] placed Tettigometridae in a more nested position in the tree, and this result was corroborated by an analysis based on partial *18S rDNA* sequences [8]. Recent morphological and molecular studies concur that the Delphacidae and Cixiidae are sister lineages to other fulgoroids, and Tettigometridae is more nested within the tree [9]–[12]. Despite intensive study, some major aspects of the planthopper phylogeny remain unresolved, including monophyly of some families and the interfamily relationships within Fulgoroidea.

According to the study by Metcalf [13], five subfamilies within Issidae were defined and this constitutes the classification of this family. However, recent studies using molecular evidence questioned the monophyly of Issidae [9]–[11]. In addition, the monophyletic Nogodinidae remains controversial [10], [11], [14]. While some taxa were proposed to be subvided, others were favored to be combined. For example, Fennah [15] considered acanaloniids as subfamilies of Issidae. Similarly, based on the structure of antennal sensilla, Liang [16] pointed out the possibility that Achilixiidae are included in Cixiidae. As stated by Hamilton [12]: “Very few of the putative families of Fulgoroidea are clearly monophyletic” (p. 71). Therefore, further taxon sampling and new characters are needed to test the monophyly of these families.

At present, the fossil record for fulgoroids is very incomplete. The earliest Fulgoromorpha fossil record is found in deposits dating to the mid-Late Permian (260 Mya) [17]. However, planthoppers are then scarce until the Jurassic period (ca. 210 Mya) [18], and the Jurassic/Cretaceous boundary and Cretaceous period were important times for diversification of extant Fulgoromorpha [19]. Mesozoic fossil beds with numerous Fulgoroidea preserved in whole-bodied condition only contained members of families Cixiidae, Achilidae, probable Derbidae, and Fulgoridae [19]. Although the data are scarce, estimation of divergence dates among living planthoppers could provide some insights into the evolution of Fulgoroidea.

Molecular phylogenetic analyses concerning the superfamily Fulgoroidea have been based solely on either nuclear [8], [11] or mitochodrial [9], [10] markers. These molecular investigations clearly confirmed the sister position of Delphacidae-Cixiidae to other families and the more nested Tettigometridae, but evidence for monophyly of Fulgoroidea as well as for the family-level affiliations of planthoppers is still lacking. Nuclear and mitochondrial genomes have different modes of inheritance, and the effectiveness of nuclear loci and of mitochondrial DNA for tracking phylogeny may differ among phylogenetic levels. Comparative studies have shown that nuclear markers are better suited for inferring deep arthropod relationships, as the mitochondrial genome is generally more saturated, compositionally biased towards adenine and thymine, and evolves at a much faster rate than the nuclear genome [20], [21]. Thus, knowing the specific limits for each set of nuclear or mitochondrial markers, and conducting molecular phylogenetic analyses based on separate or combined analysis of multiple loci may be useful in elucidating the evolutionary relationships of Fulgoroidea.

In this paper, we expanded upon a recent phylogenetic study by adding more sequences and new taxa. This is the first comprehensive analysis incorporating both nuclear (*18S* and *28S*) and mitochondrial (*16S* and *cytb*) markers into the phylogenetic reconstruction of Fulgoroidea. Additionally, we tentatively provide divergence date estimates based on the concatenated dataset.

## Materials and Methods

### Molecular Markers and Taxon Sampling

To provide a robust phylogenetic estimate for Fulgoroidea, we analyzed an expanded dataset including a larger number of *18S* sequence data from some genera not included in the analysis of Urban and Cryan [11]. Additionally, we incorporated nuclear *28S* and two additional gene segments. Both of these added genes are maternally transmitted: the mitochondrial *16S* ribosomal DNA and *cytb*. Some sequences were acquired directly from GenBank, while others were newly produced in this study. The *18S* sequence dataset includes the most complete taxon sampling, which represents 133 ingroup species from 110 genera in 19 families in Fulgoroidea. The *28S* dataset includes 57 ingroup species representing 39 genera in 18 families, *16S* for 44 ingroup species representing 31 genera in 15 families, and *cytb* for 44 ingroup species representing 30 genera in 14 families. Sixteen other hemipteran species related to Fulgoroidea were selected as outgroups for the *18S* dataset. Due to missing data, the outgroup number varied among datasets. Table S1 gives detailed information for all samples used.

All adult specimens were morphologically identified, and preserved in 100% ethanol and stored at −80°C in the Key Laboratory of Animal Evolution and Systematics, Institute of Zoology, Chinese Academy of Sciences.

### DNA Extraction, PCR Amplification and Sequencing

Total genomic DNA extraction was performed according to Aljanabi and Martinez [22], where thoracic and leg muscle tissues were used. The head and abdomen were stored in 100% ethanol as primary voucher.

Two mitochondrial and two nuclear DNA markers were targeted for each sample. Sections of the large subunit *16S* ribosomal DNA (*16S*) and cytochrome b (*cytb*) genes were amplified using primers revised from Simon et al. [23]. The partial sequences of nuclear large subunit *28S* ribosomal DNA (*28S*) and small subunit *18S* ribosomal DNA (*18S*) were obtained using primers designed for the present study. Oligonucleotide primers used in polymerase chain reactions (PCRs) are listed in Table 1, and were synthesized at Invitrogen by Life Technologies (China). PCRs were made in a 25 µl volume. All PCR conditions follow the standard three steps: an initial denaturation step of 5 min at 94°C, followed by 35 cycles of a 50 s denaturation at 94°C, a 50 s annealing at 50–60°C, and a 1–3 min elongation at 72°C, followed by a 10 min final elongation step at 72°C. The PCR products were electrophoretically inspected in 1.5% agarose gels, and directly sequenced after purification. DNA sequencing was performed with a BigDye Terminator Cycle Sequencing Kit and an ABI 3730XL Genetic Analyzer (PE Applied Biosystems, USA). All fragments were sequenced in both directions. GenBank accession numbers for all sequences newly obtained in this study are JX556694–JX556864 and KC517496 (Table S1).

**Table 1:** Primers used to amplify and sequence two nuclear genes and two mitochondrial genes.

Up primers	Sequence (5′→3′)	Down primers	Sequence (5′→3′)
Ful_18S_F	GAGAAACGGCTACCACATC	Ful_18S_R	GTCCGAAGACCTCACTAAAT
Ful_28S_F	AACAGCCGTTGCACAAGA	Ful_28S_R	GGACACCTGCGTTATCATTT
Ful_16S_F	CCGGTTTGAACTCAGATCATGTAA	Ful_16S_R	ATTTATTGTACCTTTTGTATCAG
Ful_cytb_F	GTTCTACCTTGAGGTCAAATATC	Ful_cytb_R	TTCTACTGGTCGTGCTCCAATTCA

### Sequence Alignment and Analyses

Raw sequence files were proofread and aligned into contigs in BioEdit version 7.0.5.3 [24]. Contig sequences were checked for ambiguous base calls, and only non-ambiguous regions were used for analyses. BLAST searches were conducted for each sequence to ensure its identification. All sequence alignments were performed automatically using Clustal W and MUSCLE as implemented in MEGA 5 [25] with default options, and further optimized by eye. Compared with Clustal W, MUSCLE achieved more accurate alignments, especially for the *18S* dataset. Accordingly, we preferred the MUSCLE alignments. The protein-coding gene *cytb* could be unambiguously aligned against the aligned amino acid sequences with no indels. Ambiguously aligned regions in *18S*, *28S* and *16S* were excluded from the analysis.

Nucleotide statistics and sequence analysis were performed in MEGA 5 [25] on all sequences for each gene segment. Homogeneity of base frequencies across taxa was tested using PAUP* 4.0b10 [26]. Potential saturation in the protein coding gene *cytb* was assessed by plotting transitions and transversions for each codon position against genetic distance using DAMBE 5.1.2 [27].

### Phylogenetic Analyses

The separate and combined datasets were used for phylogenetic analysis by maximum likelihood (ML) and Bayesian inference (BI). In view of the nucleotide saturation in the mitochondrial genes, the *cytb* sequences were translated into amino acid sequences using the invertebrate mitochondrial genetic code. Thus, five datasets were used in phylogenetic analyses: *18S*, *28S*, *16S*, *cytb* (amino acid sequences), and a combined dataset (both nuclear and mitochondrial data). The most appropriate substitution model for each nucleotide sequence dataset was selected using the Akaike Information Criterion as implemented in MrModeltest v2.3 [28]. For protein sequences, the substitution model was selected by ProtTest v3.0 [29].

In the ML analyses, tree searches with each dataset were performed under the best models using software PhyML v 3.0 [30]. Support for nodes was estimated by analyzing 1000 bootstrap pseudoreplicates.

BI analyses were conducted in MrBayes 3.2 [31] with the following options: independent substitution model for each partition, four Markov chains, two independent runs each for 15–25 million generations, sampling every 1000th generation, and with the first 25% discarded as burn-in. Stationarity was considered to be reached when the average standard deviation of split frequencies fell below 0.05. In addition, the Potential Scale Reduction Factor was used as a convergence diagnostic. We used the posterior probability (PP) of each node to estimate support.

### Hypothesis Testing

Hypothesis testing was done in a maximum likelihood framework using the concatenated dataset. Based on the new results obtained in the current study, we tested several alternative positions for some interesting groupings or uncertain branching relationships (Table 2). Additionally, different phylogenetic hypotheses formulated from prior morphological [4], [5] or molecular [7], [11] analyses were tested against the combined ML tree obtained with PhyML. The alternative constrained topologies were reconstructed using the program Garli 2.0 [32]. The sitewise log-likelihoods were calculated under the GTR+I+G model for each topology in PAUP* and used as input for CONSEL 0.1f [33]. Both the Shimodaira-Hasegawa test [34] and the Approximately Unbiased test [35] were performed.

**Table 2:** Alternative phylogenetic hypotheses tests (*and ** indicate significance at the 5% and 1% level).

Hypothesis	Item	Rank	*P*-value	
			SH	AU
ML (No constraint enforced)	1	1	0.978	0.732
monophyly of Fulgoroidea	2	2	0.978	0.732
(Delphacidae and, Cixiidae) as sister group to the rest of Fulgoroidea	3	3	0.978	0.732
Tettigometridae as the clade branching off first in Fulgoroidea	4	10	0.677	0.035^*^
monophyly of Lophopidae, Eurybrachidae	5	6	0.938	0.566
Lophopidae sister to Eurybrachidae	6	7	0.938	0.566
Flatidae sister to Ricaniidae	7	5	0.978	0.732
Caliscelidae sister to Tettigometridae	8	9	0.836	0.433
((Achilidae, Achilixiidae),Derbidae)	9	12	0.504	0.046^*^
Kinnaridae sister to Meenoplidae	10	11	0.601	0.083
Acanaloniidae sister to Issidae	11	8	0.429	0.954
Fulgoridae sister to Dictyopharidae	12	4	0.978	0.732
Asche (1987)	13	16	0.000	6e−054^**^
Emeljanov (1990)	14	15	0.000	3e−052^**^
Bourgoin (1993)	15	14	0.000	0.001^**^
Urban and Cryan (2007)	16	13	0.000	0.001^**^

The “Hypothesis” column indicates the constraints introduced in the phylogenetic analysis. The “Rank” column shows the order of each constraint compared with the ML tree inferred from our combined dataset. *P*-values are given for the Shimodaira-Hasegawa (SH) and approximately unbiased (AU) tests.

### Divergence Date Estimation

The dating analysis based on combined dataset was performed under the GTR+I+G substitution model using BEAST 1.7.1 [36]. The priors for the mean and standard deviation of the ingroup root age were set to 260 million years and 10 million years, respectively [17]. We used a relaxed molecular clock with the uncorrelated log-normal model [37] and a Yule speciation model for the tree prior. Two independent Markov chain Monte Carlo (MCMC) runs were performed each for a total of 20 million generations (10% burnin) sampled every 1000 steps. Tracer 1.5 [38] was used to check MCMC convergence. The BEAST maximum clade credibility chronogram was visualized in FigTree 1.3.1 [39].

## Results

### Sequence Characteristics

The number of taxa included in the separate *18S* analysis was 149, which included 16 outgroups. The combined dataset contained 71 sequences of *18S*, with 65 for the ingroup and 6 for the outgroup. Using BLAST searches in the NCBI database, we found above 80% similarity for *18S* between some species sequenced in this study and other organisms (e.g., 86% identities between *Lycorma delicatula 18S rDNA* and *Homo sapiens* RNA-RN18S1). After alignment, and removal of ambiguously aligned sites, 1321 bp nucleotide sequences of *18S* were used for tree reconstruction. For the combined dataset, sequences of the nuclear locus *28S* were obtained for 60 taxa, with missing data due to failed PCR amplifications or absence in Genbank. The final *28S* alignment consisted of 1306 nucleotide positions, which contained 719 variable sites and 469 parsimony-informative sites. For mitochondrial genes, we obtained a total of 1085 bp, including 588 bp of *cytb* with no indels, no premature stop codons and no ambiguous base calls, and 497 bp of *16S*. The two mitochondrial gene fragments contained 734 parsimony-informative sites. A summary of the markers used in this study is presented in Table 3.

**Table 3:** Summary of markers used in the combined analysis.

Loci		Length (bp)	New sequences obtained		SequencesfromGenBank		Total number of sequences	Conserved sites	Variable sites	Parsim-Info sites
*18S*		1321	45		26		71	781	540	332
*28S*		1306	39		21		60	587	719	469
*16S*		497	44		7		51	100	397	346
*cytb*										
	1st	196	−		−		−	63	133	119
	2nd	196	−		−		−	82	114	79
	3rd	196	−		−		−	0	196	190
	1st+2nd	392	−		−		−	145	247	198
	All	588	44		7		51	145	443	388
		**Nucleotide composition**								
		**T**		**C**		**A**	**G**	**% A+T**	**χ^2^**	**P**
*18S*		24.23		24.75		21.95	29.07	46.18	55.01	1.000
*28S*		20.65		27.01		20.64	31.70	41.29	72.09	1.000
*16S*		32.05		16.43		43.00	8.52	75.05	376.80	0.000
*cytb*	1st	30.1		15.82		38.27	15.82	68.37	111.65	0.992
	2nd	45.92		23.47		20.41	10.20	66.33	31.85	1.000
	3rd	37.25		9.69		49.49	3.57	86.73	403.84	0.000
	1st+2nd	38.01		19.64		29.34	13.01	67.35	87.40	1.000
	All	37.76		16.33		36.05	9.86	73.81	240.94	0.000
		**Saturation test**								
		**Iss**	**Iss.cSym** a			**Psym** b	**Iss.cAsym** c	**Pasym** d		
*18S*		0.038	0.699			0.0000	0.373	0.0000		
*28S*		0.058	0.713			0.0000	0.385	0.0000		
*16S*		0.421	0.702			0.0000	0.377	0.1290		
*cytb*	1st	0.309	0.697			0.0000	0.390	0.0477		
	2nd	0.185	0.697			0.0000	0.390	0.0000		
	3rd	0.720	0.697			0.4335	0.389	0.0000		
	1st+2nd	0.246	0.687			0.0000	0.358	0.0000		
	All	0.372	0.707			0.0000	0.379	0.7658		

a Index of substitution saturation assuming a symmetrical true tree.

b Probability of significant difference between Iss and Iss.cSym (two-tailed test).

c Index of substitution saturation assuming an asymmetrical true tree.

d Probability of significant difference between Iss and Iss.cAsym (two-tailed test).

A chi-square test for base compositional homogeneity revealed significant heterogeneity among taxa for the combined dataset (p<0.0001). To detect the source of this heterogeneity within the data, all loci and each codon position of *cytb* were tested individually. We found that the base composition in *16S* and the 3rd codon positions of *cytb* varied significantly (Table 3), with both regions exhibiting great A+T bias (>70%).

Because saturation in substitutions can lead to confusing effects on phylogenetic inferences [40], the level of saturation in each gene partition was explored (Table 3). We first calculated an index of substitution saturation (Iss) and tested it with standard statistical tests against critical values (Iss.c) using DAMBE [41]. No saturation was detected in the *18S*, *28S* and *16S* alignments (Iss significantly<Iss.c). For the 3rd codon positions of *cytb*, little saturation was detected, with the resulting Iss (0.720) marginally higher than Iss.cSym (0.697). This means that the sequences may still be useful under the assumption of a symmetrical tree topology. However, the Iss values were significantly higher than Iss.cAsym (0.389), indicating a poor phylogenetic signal if the true topology is very asymmetrical [42]. Taking into account the possible influences caused by saturation in substitutions and the base compositional heterogeneity described above, we estimated trees using the amino acid sequences of *cytb*.

### Model Selection

The results indicated that GTR+I+G is the best-fit nucleotide substitution model for *18S*, *28S*, *16S*, and the combined dataset as proposed by MrModeltest. However, because the parameter “I” (proportion of invariant sites) is sensitive to the number and divergence of sequences included in the data set [43], we conducted phylogenetic analyses under the GTR+G model. mtArt+G+F was selected for the *cytb* amino acid dataset by ProtTest.

### Separate Analyses

The separate analyses of *18S* and *cytb* resolved several of the higher-level relationships within Fulgoroidea (Figure S1 and Figure S2). ML analysis of the *18S* dataset recovered Fulgoroidea as monophyletic with good support (BS = 100), with Delphacidae and Cixiidae placed as the sister lineage to the remaining families; Tettigometridae was nested within a large clade which also included Achilixiidae, Achilidae, Kinnaridae, and Meenoplidae; Kinnaridae was recovered as sister to a monophyletic Meenoplidae; Lophopidae and Eurybrachidae were grouped together; and Dictyopharidae and Fulgoridae were grouped together. The independent Bayesian analysis of *18S* only recovered the grouping of Delphacidae and Cixiidae as the sister lineage to other families in Fulgoroidea, but the relationships of the remaining taxa were poorly resolved (data not shown).

For the *cytb* amino acid sequences, both ML and BI analyses achieved better resolution of the relationships in Fulgoroidea. The ML analysis of *cytb* retrieved a monophyletic Fulgoroidea, and the placement of Delphacidae and Cixiidae as the sister group to all other families. In addition, several sister relationships were recovered: Lophopidae and Eurybrachidae, Flatidae and Ricaniidae, and Dictyopharidae and Fulgoridae. Overall, *cytb* provided strong support (BS >80, PP>0.9) for several shallow nodes, but low support (<70) for most deep nodes.

The trees estimated from *28S* and *16S* were much less resolved, compared with *18S* or *cytb*. This may be due to much more ambiguity in the sequence alignments of *28S* and *16S*, resulting in poor phylogenetic information for tree reconstruction.

### Combined Analysis

By combining all nuclear and mitochondrial data, we obtained a well-supported phylogenetic hypothesis for Fulgoroidea. Bootstrap support and posterior probabilities are high for almost all nodes. Moreover, shallow nodes were better resolved by the combined dataset than individual *18S* analysis, and for the deep nodes better than *cytb*. Thus, we consider the combined ML tree to be a very strongly supported topology (Fig. 1), and our best current estimate of the phylogeny of Fulgoroidea. Below we focus on this tree unless otherwise stated. Bayesian analysis of the combined dataset recovered similar relationships to ML (Fig. 2). However, except for the position of Delphacidae and Cixiidae in Fulgoroidea, the Bayesian tree was less resolved than the ML tree.

**Figure 1:** Maximum-likelihood tree estimated from the combined datatset of 65 taxa of Fulgoroidea. Values above branches denote ML bootstrap support (≥70). The red numbers in circles correspond to ten major clades discussed in the text.

**Figure 2:** The 50% majority-rule consensus tree estimated from the Bayesian analysis based on the combined dataset. Values above branches denote posterior probabilities (≥0.9).

As with *18S* or *cytb*, our combined data analyses confirmed a well-supported monophyletic Fulgoroidea. Cixiidae and Delphacidae were consistently placed as the sister group to all other families. The monophyletic Kinnaridae and Meenoplidae were the sister group to the remaining families. Although the sister relationship between Kinnaridae and Meenoplidae was recovered, the support for this relationship was relatively low (BS <50). Clade 3 included one representative of Lophopidae and the family Eurybrachidae. Clade 4 contained the rest of Fulgoroidea, which comprised two major groups. One consisted of clades 5, 6, and 7, while the other contained clades 8, 9, and 10.

Clade 5 was composed of Flatidae and Ricaniidae. These formed a well-supported sister group (BS = 95). Clade 6 included the families Achilidae, Tropiduchidae and part of Nogodinidae. Among these, Tropiduchidae and part of Nogodinidae were recovered as sister groups. Part of Nogodinidae, part of Lophopidae, the family Caliscelidae and the Tettigometridae composed Clade 7. Of these, Caliscelidae and Tettigometridae were retrieved as sister groups.

The representative of Achilixiidae, part of Nogodinidae, and the family Derbidae constituted the sister clade to all others in the second major group. Clade 9 was a monophyletic and strongly supported lineage that comprised Dictyopharidae and Fulgoridae. The sister grouping of Fulgoridae and Dictyopharidae was consistently recovered in both inference methods. The remaining species made up Clade 10, which included Acanaloniidae and Issidae. Acanaloniidae was the sister family to Issidae.

### Hypothesis Testing

Alternative hypotheses were compared based on previous studies or unstable branching in the present analyses. Results of comparisons are summarized in Table 2. In both Shimodaira-Hasegawa (SH) and approximately unbiased (AU) tests, the phylogenetic tree inferred by ML analysis of the combined dataset has a very high probability (SH 0.978, AU 0.732), and the hypothesis of monophyletic Fulgoroidea received the same probabilities. This further confirmed that our data strongly supported the monophyly of Fulgoroidea. The position of Delphacidae and Cixiidae as the sister group of the remaining Fulgoroidea was also corroborated. Instead, the AU test rejected placement of Tettigometridae as the sister family to the remaining taxa within Fulgoroidea (*p*<0.05). In addition, the topology assuming both Lophopidae and Eurybrachidae to be monophyletic was accepted statistically (*p*>0.05). Several sister-group relationships were determined: Lophopidae and Eurybrachidae, Flatidae and Ricaniidae, Fulgoridae and Dictyopharidae, and Kinnaridae and Meenoplidae. The sister relationship between the grouping of Achilidae and Achilixiidae with Derbidae was rejected by the AU test, but not by the SH test. This suggested that the SH test was generally more conservative than the AU test.

The alternative hypotheses from previous studies were all rejected by SH and AU tests. Nevertheless, the results of the “Rank” generated by CONSEL clearly showed that our preferred topology was more similar to previous molecular studies than to those based on morphology (Table 2).

### Divergence Dates

Divergence time estimates are illustrated in Fig. 3. This maximum credibility tree generated by BEAST was comparable to that produced by PhyML. The key nodes had high posterior probabilities, including the placement of Cixiidae and Delphacidae. The total ingroup was estimated to have shared a common ancestor around 255 Mya (215–293 Mya), which was similar to the fossil evidence [18]. The divergence time of Cixiidae and Delphacidae was around 221 Mya. Tettigometridae appeared later, at approximately 65 Mya. The split of the achilid clade from other fulgoroids was estimated to be about 133 Mya, a date congruent with the fossil record [44]. The lineages comprising the representatives of Ricaniidae diverged around 98 Mya (95% highest posterior density intervals: 60∼138 Mya) in the Late Cretaceous, which was older than previous studies [45].

**Figure 3:** Chronogram of Fulgoroidea estimated using the Bayesian phylogenetic software BEAST. Time units are in millions of years before present. Estimated divergence times are shown near nodes, while blue bars represent 95% credibility intervals. The values on the branches denote the posterior probabilities (≥0.9).

## Discussion

Fulgoroidea is of economic importance, because many species in this group are pests on agricultural crops. However, the relationships among the main lineages of the Fulgoroidea are poorly understood, and previous analyses yielded conflicting hypotheses. Even the family-level classification of Fulgoroidea has remained controversial. As mentioned by Bourgoin et al. [8]: “…that currently available phylogenies of family level affiliations within Fulgoromorpha are premature” (p. 219). A quasi-phylogenetic classification by Muir [46] is traditionally used to delimit numerous families within Fulgoroidea. However, the monophyly of Fulgoroidea is not evident, and many interfamily relationships remain unresolved in recent studies [11], [12].

Our molecular study has produced a set of well-supported phylogenetic relationships based on an expanded dataset, which includes both nuclear and mitochondrial sequences for the main clades. Phylogenetic analysis of *18S* strongly supported monophyly of Fulgoroidea, while separate analyses of *28S*, *16S* and *cytb* did not provide such support. Combined analysis of all four genes recovered a consistent, well supported, monophyletic Fulgoroidea across methods of tree reconstruction (BS = 100, PP = 1.0). The support for monophyly was greater than in analyses of individual genes. In addition, the combined analyses resolved the monophyly of some families: Cixiidae, Delphacidae, Ricaniidae, Dictyopharidae, and Fulgoridae. All these families were confidently recovered as monophyletic (BS >75, PP>0.95).

### Phylogenetic Relationships within Fulgoroidea

Several previous morphology-based studies using a largely unstable character set (e.g., wing morphs, and the position of the median ocellus) have resulted in different topologies for planthoppers. The influential classification by Muir [46] used the structure of the aedeagus, which is a character of extreme variability. Similarly, other earlier studies were mainly based on the features of the male genitalia [4], [5]. Fulgoroidea has the synapomorphic characters of antennal sensillae and hind coxae, as mentioned as long ago as 1890 by Hansen [3], [47], with such non-homoplastic morphological characters being the best test of monophyly. Recent genetic studies of Fulgoroidea confirmed some of the classifications inferred from morophological characters, but simultaneously cast doubt on the presumed affinities of many genera or families.

Basal branching patterns have been the focus of past studies of the phylogeny of Fulgoroidea. Due to morphological characters shared with Cicadoidea, Tettigometridae had been treated as the sister lineage to all other families within Fulgoroidea by Muir [3]. Thereafter, this proposed position of Tettigometridae was strengthened by several studies based on non-cladistic analyses of morphological characters [4]–[6]. However, Bourgoin [8] suggested that the morphological characters supporting the placement of Tettigometridae were subject to convergence, and he recovered the cixiid and the delphacid lineages as the sister group to all other fulgoroids based on *18S* rDNA. Three subsequent studies based on molecular data supported this placement of Cixiidae and Delphacidae [10], [11]. Based on morphological data, the relationship between Cixiidae and Delphacidae is difficult to resolve, because these two families share extensive plesiomorphic characters. Muir [3] proposed that Delphacidae arose from within Cixiidae [3]. Nevertheless, Asche [4] considered Delphacidae and Cixiidae as sister families. Emeljanov [5] proposed that Cixiidae is sister to all other fulgoroids except Tettigometridae. Based mainly on antennal characters, Delphacidae was inferred as the sister group to all other families by Hamilton [12], with Cixiidae being sister to the ingroup families. Our findings are consistent with those of Urban and Cryan [11] showing that Cixiidae is sister to Delphacidae and that together they form the sister group to all other families in Fulgoroidea [11].

The ML analysis of the combined dataset recovered the grouping of Kinnaridae and Meenoplidae as the sister group to all fulgoroids excluding Cixiidae and Delphacidae. In previous studies, Kinnaridae was assigned as a sister group to Meenoplidae [5], [7], [11]. Our results presented here are congruent with theirs. The prominent genal lobes and distinctive nymphal traits associate Lophopidae with Eurybrachidae [12]. Some analyses based on morphological or molecular characters recovered Lophopidae and Eurybrachidae as sister groups [5], [11]. However, a morphology-based study suggested that Lophopidae was not a monophyletic lineage: two South American genera were always recovered outside the major lophopid clade [48]. Yet, it still supported Eurybrachidae as the sister group of Lophopidae [48]. Our *18S* dataset also grouped these two families together. In our analyses of the combined dataset, the Bayesian tree grouped Lophopidae and Eurybrachidae together with Lophopidae being paraphyletic, and the ML tree also failed to retrieve a monophyletic Lophopidae. However, our hypothesis tests could not rejected the monophyly of Lophopidae and the sister relationship between Lophopidae and Eurybrachidae. We believe that limited taxon sampling of Lophopidae and lower sequence homology may have led to this unexpected result.

The sister relationship between Ricaniidae and Flatidae was strongly supported by the concatenated dataset with different analytical methods. Although this sister relationship is a novel placement inferred from molecular data, morphological evidence supporting this arrangement has been noted by previous authors [5], [7]. Loss of posterior tentorial arms has been interpreted as shared derived characters between Ricaniidae and Flatidae [7]. The recovery of this lineage is also consistent with the findings of Asche [4], implying that both Flatidae and Ricaniidae have a piercing-excavating ovipositor.

Most of the previous morphological studies have proposed a close relationship between Achilixiidae and Achilidae. Though Urban and Cryan [11] could not retrieve these two groups in one clade, their results showed a closer relationship of Achilixiidae to Achilidae [11]. In contrast, our ML analysis of the concatenated dataset did not support the closer relationship of Achilixiidae to Achilidae. Our Bayesian analysis recovered Achilixiidae as the sister family to Achilidae, but the posterior probability for this node was lower than 0.50. Based on studies of external morphology of antennal sensilla, Liang [16] considered the basal flagellar process as an apomorphy of Achilixiidae and Cixiidae, and suggested that two achilixiid subfamilies (Achilixiinae and Bebaiotinae) should be moved to Cixiidae. Further comparative morphological and molecular research on the phylogenetic position of Achilixiidae is necessary, especially with more species representing achilixiids.

Monophyly of Tropiduchidae was supported by different methods (BS = 100 and PP = 1.0). Among the trees generated in this study, Tropiduchidae and partial Nogodinidae always clustered together. In previous studies, the exact relative phylogenetic position of Tropiduchidae remained uncertain [11]. Yeh et al. [9] suggested that Tropiduchidae had a closer relation to Flatidae. The molecular analyses of Urban and Cryan [11] showed that Tropiduchidae was the sister lineage to some lineages of Nogodinidae, which is similar to our findings.

The placement of Tettigometridae among higher Fulgoroidea was decisively demonstrated by our data and has been corroborated by other genetic studies [8], [10], [11]. A recent morphological analysis yielded a similar placement of Tettigometridae [12]. In the present analysis, the monophyletic Caliscelidae was always retained and more distantly related to other issids. Caliscelidae and Tettigometridae were placed as sister taxa in the ML analysis of the combined dataset. These data are congruent with the proposal to raise Caliscelinae to family status, and we can therefore confirm the paraphyly of Issidae. Nevertheless, the new placement of Caliscelidae (as the sister group to tettigometrids) is only tentatively proposed due to lower support (BS <70).

Fossil evidence shows that Derbidae may be a group branching off early in Fulgoroidea [19]. However, except for the ML analyses of *18S*, our other datasets placed Derbidae in a more nested position in the phylogeny. Urban and Cryan [11] suggested that Derbidae has a closer relationship to Achilidae or Achilixiidae. Although this sister relationship was not retrieved in the current study, our data did not reject this arrangement (*p*>0.05 in SH and AU tests).

Morphologists agree that Fulgoridae is a sister group to Dictyopharidae, because both lineages share distinctive male genitalia structure [4], [5], [7], [46]. Our phylogenetic analyses that combined mitochondrial and nuclear data also strongly supported such a grouping.

The monophyly of Issidae has been questioned by previous studies [5], [9]–[11], [49]. Emeljanov ([49] raised the issid subfamily Caliscelinae to family rank. Based on the analysis of some morphological features, Yang and O’Brien [10] also proposed that Caliscelinae should be raised to a separate family Caliscelidae. Furthermore, several molecular studies unambiguously rejected the monophyly of Issidae, placing Caliscelinae outside Issidae [10], [11]. Our analyses also affirmed Issidae to be non-monophyletic. In our ML analysis of the combined dataset, however, we inferred that Acanaloniidae has a closer relationship to Issidae. This result is consistent with some morphological analyses [4], [5], [7], but is in contrast with others [11], [49].

### Divergence Time Estimation

The superfamily Fulgoroidea started to diversify in the mid-Late Permian (260 Mya), and their presumed ancestors, Coleoscytoidea, extended back into the mid-Permian (270 Mya) [17]. From our analyses, Fulgoroidea began to diverge in the Late Permian, with further diversification at the family level lasting from the Late Triassic to the Early Cretaceous (Fig. 3). Within Fulgoroidea, the first fossils of Cixiidae have been dated to the beginning of the Jurassic period (210 Mya) [18], followed by fossils of Achilidae (135 Mya) [44]. In addition, the oldest fossil known for Ricaniidae does not appear until the Palaeocene (<65 Mya) [45]. Our molecular date estimates suggest that most species of Fulgoroidea underwent a relatively rapid radiation during the Jurassic and Cretaceous, which is consistent with the findings of Szwedo et al. [50]. Additionally, both studies are consistent with respect to basal relationships within Fulgoroidea. Cixiidae and Delphacidae were placed as the sister lineage to all other families. The lineage Cixiidae could be traced back into the Early Jurassic (195 Mya), while Delphacidae diverged in the Early Cretaceous (around 129 Mya). Although the congruence between date estimates and fossil evidence provides some support in the reconstructed phylogeny of Fulgoroidea, Bayesian analysis using BEAST yielded an older origin for some fulgoroid groups. This is consistent with the idea that molecular estimates should be earlier than fossil ages. Nevertheless, the fossil evidence for Fulgoroidea is scanty at present. Thus, our divergence date estimates should only be regarded as provisional. In future studies, it will be important to explore correlations with historical biogeography and with morphological trait evolution. Support for our date estimates needs more fossil, morphological, or molecular evidence.

### Conclusion

Our ML analysis of combined nuclear and mitochondrial markers recovered some relationships with strong support among major lineages of Fulgoroidea, but our Bayesian analysis only resolved the basal relationships reliably. Individual analyses of nuclear *18S* and mitochondrial *cytb* showed the utility of these two markers in elucidating relationships among fulgoroids. Although the phylogenetic analyses presented here provide a robust hypothesis for the higher-level relationships within Fulgoroidea, further investigations are necessary to fully understand the evolution of planthoppers. Because Fulgoroidea is such a highly diverse insect group, our taxon sampling is sparse. Thus, relationships reconstructed in this paper are still tentative. Further research is required with greater sampling and with more molecular and morphological characters.

## Supporting Information

Figure S1 **Maximum-likelihood tree estimated from the** ***18S*** **dataset of 133 fulgoroid species.** ML bootstrap values (≥70) are shown behind the nodes.
(ZIP)

Figure S2 **Trees estimated from the** ***cytb*** **datatset of 44 fulgoroid species.** (A) Maximum likelihood analysis. (B) Bayesian analysis. ML bootstrap values (≥70) and Bayesian posterior probabilities (≥0.9) are presented.
(ZIP)

Table S1 **Taxa sampled.**
(ZIP)
